# Bailing Capsule combined with α-ketoacid tablets for stage 3 chronic kidney disease: Protocol of a double-blinded, randomized, controlled trial

**DOI:** 10.1097/MD.0000000000025759

**Published:** 2021-05-21

**Authors:** Xiuhong Hu, Jing Wang, Hongjuan Yang, Suhua Ji, Yuhong Li, Baozhen Xu, Hongrui Cui

**Affiliations:** The First Hospital of Hebei Medical University, Shijiazhuang, Hebei Province, China.

**Keywords:** Bailing capsule, Chinese patent medicine, chronic kidney disease, kidney function, protocol

## Abstract

**Background:**

Chronic kidney disease (CKD) is a progressive and irreversible loss of kidney function. After stage 3, there will be increased risks of hypertension, heart failure, bone disease, anemia, gastrointestinal symptoms, and progression to end-stage kidney failure without proper intervention and treatment. Compound α-ketoacid tablets (KA) administration plays an important role in clinical CKD adjunctive therapy for patients with restricted protein intake. Bailing Capsule (BC), a commonly used Chinese patent medicine for renal diseases, could regulate human immune function, repair renal tubular epithelial cells, prevent renal tubular atrophy, and reduce kidney damage to improve renal function. In this study, we try to conduct a double-blinded, randomized, controlled trial to observe the efficacy and safety of BC combined with KA in treating patients with stage 3 CKD.

**Methods:**

This is a double-blinded, randomized, controlled trial. Patients will be randomly divided into treatment group (BC and KT) and control group (BC-simulation and KT) in a 1:1 ratio according to random number table. The treatment course will be 8 weeks, and the changes of subjective symptoms, patient global assessment (PGA) scale, serum creatinine, cystatin C, and estimated glomerular filtration rate, all related adverse events, vital sign measurements, and physical examinations will be recorded. SPSS 21.0 will be used for data analysis.

**Conclusions:**

The results will show whether BC combined with KA could alleviate the symptoms of fatigue, anorexia, halitosis, nausea, itching, and edema, improve kidney function in patients with CKD at stage 3.

**Trial registration:**

OSF Registration number: DOI 10.17605/OSF.IO/24AJ7.

## 1 Introduction

Chronic kidney disease (CKD) is a progressive and irreversible loss of kidney function, with an increased prevalence in recent years.^[1,2]^ It is mainly caused by diabetes, hypertension, and glomerulonephritis.^[3,4]^ Initially, the symptoms of CKD are insidious and then presented with fatigue, swelling legs, dizziness, and loss of appetite gradually. After stage 3, the above symptoms become more obvious, with increased risks of hypertension, heart failure, bone disease, anemia, gastrointestinal symptoms, and a progress to end-stage kidney failure without proper intervention and treatment.^[5,6]^

At present, the main principles for CKD are treating original diseases, low-protein diet, essential amino acids intake, and management of complications. Although it could slow down the damage to kidney function, long-term low-protein diet can aggravate malnutrition in patients. Compound α-ketoacid tablets (KA) administration plays an important role in clinical CKD adjunctive therapy for patients with restricted protein intake.^[7,8]^ With appropriate proportioned essential amino acids, KA could promptly meet the needs of human synthesis to improve the protein metabolism disorder. In addition, KA could reduce insulin resistance and increase esterase activity, thereby improving patients’ glucose and lipid metabolism.

In China, Bailing Capsule (BC) is a commonly used Chinese patent medicine for renal diseases.^[9,10]^ It is composed of Cordyceps mycelium, which is rich in a variety of trace elements, amino acids, adenosine, and cordycepin to improve blood circulation, inhibit neurotransmitter release and regulate adenylate cyclase activity. Studies have shown that BC could regulate human immune function,^[11–13]^ repair renal tubular epithelial cells, prevent renal tubular atrophy, and reduce kidney damage to improve renal function.^[14,15]^ Our group tried to use the combination of BC and KA to treat CKD patients, and we preliminarily found the therapy could improve the symptoms of fatigue and dizziness to improve the quality of life. However, there are few highquality studies to observe the efficacy of BCs and α-ketoacid tablets in the treatment of stage 3 CKD. In this study, we try to conduct a double-blinded, randomized controlled trial to observe the efficacy and safety of BC combined with KA in treating patients with stage 3 CKD.

## 2 Methods

### 2.1 Study design

From June 1st, 2021 to May 31st, 2022, the double-blinded, randomized controlled trial with a registration number of DOI 10.17605/OSF.IO/24AJ7 will be conducted in the First Hospital of Hebei Medical University. The trial has been approved by the Health Research Ethics Board in the hospital. The procedure will be in accordance with the Declaration of Helsinki. The study design is shown is Figure 1.

**Figure 1:** Flow diagram of the study.

### 2.2 Patients

CKD patients referring to the First Hospital of Hebei Medical University will be assessed for screening. Before randomization, a written informed consent will be signed for all the patients or or authorized persons, and they are free to discontinue the trial at any time.

The inclusion criteria are as follows:

1. aged 18 to 80 years’ old;
2. CKD in stage 3 (30 mL/min/1.73 m^2^<estimated glomerular filtration rate<59 mL/min/1.73 m^2^);
3. with written informed consent.

The exclusion criteria are as follows:

1. with a history of allergic to ingredients of BC or KA;
2. with a history of kidney transplant;
3. with uncontrolled diabetes (HbAlc) >10% and hypertension (systolic blood presuure ≥170 mmHg or diastolic blood pressure ≥100 mmHg);
4. complicated with hepatic impairment, infection, or malignant tumor;
5. women in pregnant or lactating.

### 2.3 Randomization and blinding

Patients will be randomly divided into treatment group (BC and KT) and control group (BC-simulation and KT) in a 1:1 ratio according to random number table. The physician, patients, assessors, and analysts will all be blinded to the allocation. The BC-simulation is presented in the same package, appearance, and taste with BC to maintain blinding.

### 2.4 Interventions

The same initial treatment will be applied to patients in both groups with medicines to protect the kidney, reducing blood pressure, regulating lipid. Patients will also be educated to take high-quality low-protein diet and regular exercise and rest.

In the treatment group, patients will take 2 g BCs (Hangzhou Zhongmei Huadong Pharmaceutical Co. Ltd, Z10910036) 3 times daily and 2.52 g Compound α-ketoacid tablets (Beijing Fresenius Kabi Pharmaceutical Co., Ltd, H20041442) 3 times daily simultaneously for 8 weeks.

In the control group, patients will take 2 g BC-simulations (Hangzhou Zhongmei Huadong Pharmaceutical Co. Ltd) 3 times daily and 2.52 g Compound α-ketoacid tablets (Beijing Fresenius Kabi Pharmaceutical Co., Ltd, H20041442) 3 times daily simultaneously for 8 weeks.

### 2.5 Outcome measures

The primary outcomes are the changes of subjective symptoms of fatigue, anorexia, halitosis, nausea, itching, and edema evaluated at week 0, week 4, and week 8. The corresponding score will be 2, 4, and 6, respectively, according to the degree of mild, moderate, and severe. The secondary outcomes are patient global assessment scale, serum creatinine, cystatin C, and estimated glomerular filtration rate at week 0 and 8. The patients will be followed for another 4 weeks after the treatment. The incidence and types of related adverse events, vital sign measurements, and physical examinations will also be recorded.

### 2.6 Sample size

In our preliminary study, the change of subjective symptoms in the treatment group was 7.21 ± 4.36 and 4.35 ± 3.15 in the control group. Taking α as 0.05, β as 0.2 with a 2-sided test, and considering a dropout of 20%, 72 patients will be needed totally.

### 2.7 Statistical methods

SPSS 21.0 (SPSS Inc, Chicago, IL) will be used for data analysis. The measurement data will be expressed as mean ± standard deviation. Considering the normality and homogeneity, *t* test, or nonparametric test will be applied for the changes between the 2 groups. Repeated measurement analysis of variance or generalized linear model will be applied for repeated measurement data. *P* < .05 will be considered statistically significant.

## 3 Discussion

CKD refers to chronic injury caused by various primary or secondary renal diseases, and it is characterized by insidious and slow progression. In the early stages, there are generally no symptoms or the symptoms vary with different primary diseases. Without proper intervention, it will eventually develop into uremia with the progression and the deterioration of renal function to threaten patients’ life. Therefore, it is important to effectively slow down or even halt the progression of CKD in the early stage.

Compound KA administration could function in renoprotective effect as adjunctive therapy for CKD.^[16]^ Also, it has been reported that BCs could effectively improve the kidney function in patients with nephrotic syndrome and type 2 diabetic nephropathy.^[14,15]^ Although the combination of BC and KA against CKD was rarely reported in high-quality designed trials. In this study, we try to conduct a double-blinded, randomized, controlled trial to observe whether BC combined with KA could alleviate the symptoms of fatigue, anorexia, halitosis, nausea, itching, and edema, improve kidney function in patients with stage 3 CKD. However, there are several limitations in the study. First, it is a single-centered study. Second, the study period may not be long enough to explore whether the combined treatment could delay the CKD progression.

## Author contributions

**Data collection:** Xiuhong Hu and Jing Wang.

**Data curation:** Xiuhong Hu, Jing Wang.

**Funding acquisition:** Hongrui Cui.

**Funding support:** Hongrui Cui.

**Investigation:** Suhua Ji and Yuhong Li.

**Resources:** Suhua Ji and Baozhen Xu.

**Software operating:** Jing Wang and Hongjuan Yang.

**Software:** Jing Wang, Hongjuan Yang.

**Supervision:** Yuhong Li and Baozhen Xu.

**Writing – original draft:** Xiuhong Hu and Jing Wang and Hongjuan Yang.

**Writing – review & editing:** Xiuhong Hu and Hongrui Cui.
